The article "Diagnosing Breast Cancer Based on the Adaptive Neuro-Fuzzy Inference System" was published in 2022. Journal: Comput Math Methods Med.

# Diagnosing Breast Cancer Based on the Adaptive Neuro-Fuzzy Inference System

**DOI:** 10.1155/2022/9166873

**Published:** 2022-05-11

**Authors:** S. Chidambaram, S. Sankar Ganesh, Alagar Karthick, Prabhu Jayagopal, Bhuvaneswari Balachander, S. Manoharan

**Affiliations:** ^1^Department of Information Technology, National Engineering College, Kovilpatti, 628503, Tamil Nadu, India; ^2^Department of Artificial Intelligence and Data Science, KPR Institute of Engineering and Technology, Arasur, Coimbatore, 641407, Tamil Nadu, India; ^3^Renewable Energy Lab, Department of Electrical and Electronics Engineering, KPR Institute of Engineering and Technology, Arasur, Coimbatore, 641407, Tamil Nadu, India; ^4^Departamento de Quimica Organica, Universidad de Cordoba, Edificio Marie Curie (C-3), Ctra Nnal IV-A, Km 396, E14014 Cordoba, Spain; ^5^School of Information Technology and Engineering, Vellore Institute of Technology, Vellore, 632014, Tamil Nadu, India; ^6^Department of ECE, Saveetha School of Engineering, Saveetha Institute of Medical and Technical Sciences, Chennai, Tamil Nadu, India; ^7^Department of Computer Science, School of Informatics and Electrical Engineering, Institute of Technology, Ambo University, Ambo, Post Box No.: 19, Ethiopia

## Abstract

In this work, a novel hybrid neuro-fuzzy classifier (HNFC) technique is proposed for producing more accuracy in input data classification. The inputs are fuzzified using a generalized membership function. The fuzzification matrix helps to create connectivity between input pattern and degree of membership to various classes in the dataset. According to that, the classification process is performed for the input data. This novel method is applied for ten number of benchmark datasets. During preprocessing, the missing data is replaced with the mean value. Then, the statistical correlation is applied for selecting the important features from the dataset. After applying a data transformation technique, the values normalized. Initially, fuzzy logic has been applied for the input dataset; then, the neural network is applied to measure the performance. The result of the proposed method is evaluated with supervised classification techniques such as radial basis function neural network (RBFNN) and adaptive neuro-fuzzy inference system (ANFIS). Classifier performance is evaluated by measures like accuracy and error rate. From the investigation, the proposed approach provided 86.2% of classification accuracy for the breast cancer dataset compared to other two approaches.

## 1. Introduction

Recently, data mining plays a major role in both industry and research organizations due to the accessibility of the huge volume of data and transforms these data into significant information and knowledge. Mainly classification [1] is the approach determining a classifier that compares and predict a target class with an unidentified class label. During the training phase, it follows two phases; a classifier is developed, as well as its relevant class variables. During the test phase, a set of features are applied to approximate the level of the classifier.

Before the data classification process, many preprocessing procedures have been applied. The artificial neural network (ANN) can do intellectual responsibilities like the human brain. A popular trustworthy classification method from the NN is the multilayer backpropagation network [2]. And a radial basis function [3] is a dominant neural approach that uses radial basis procedures. In that, neuron parameters are considered for producing better performance.

The artificial neural network (ANN) is a trendy data modeling approach which can carry out intelligent tasks in the same way as the human brain. ANN is well suitable for high-precision and high-learning ability purpose. One of the reliable approaches of data classification from the neural network area is the multilayer perceptron backpropagation network (MLPBPN) approach [4]. The output of this neural network technique is the linear combination of radial basis functions of inputs and neuron factors. RBFNNs helps for classification, function approximation, and prediction of time series applications.

The discrete-time linear dynamical systems [5] are used to make a spirit for the approximation. It includes time-varying systems by recurrent neural networks (RNNs). For the subclass of linear time-invariant (LTI) systems, learning a differential equation is the easiest feasible mathematical incarnation. In the experimental results, the dynamics of physical, biological, mechanical, or chemical procedures are recognized from practical input-output traces. An adaptive proportional-integral controller is used along with the proper gain variation according to the adaptive neuro-fuzzy inference system (ANFIS) to promise high performances of electric drive models with respect to the parametric differences.

In a fuzzy approach, the selected attributes are linked with a degree of membership to various groups. Both NN and fuzzy approaches are flexible to measure *I*/*O* correlations. Fuzzy systems consider figurative as well as quality-based data. The condition-oriented neuro-fuzzy approach is categorized as the linguistic fuzzy modeling that deals with the inference and fuzzy modeling technique like the Sugeno model which considers accuracy [6].

The modular neural network is an incorporation of smaller subcomplete neural network models [7]. Each model functions separately on a subportion of larger size pattern vectors. There are two ways of modularizing the neural network, i.e., modularizing learning and modularizing structure. The modular learning for pattern classification of hand-written Hindi alphabets is considered. Here, twenty-four individual subneural networks have been considered for first phase computing. Then, the collective outputs of the first phase are applied as input to the global neural network. Thus, the output of the second phase presents the desired classification of the given large training set. Neural networks of the first phase are trained locally for decomposed input patterns with gradient descent learning. Updated weights of the first phase are mapped to the global neural network. The global neural network is further trained for the collective output patterns of the first phase computing. Here, decomposition and replication concepts have been applied to perform the classification task [8].

A forecast time series model [9] is proposed which uses generalized regression neural networks. The objective is to take advantage of their inherent properties to produce fast and accurate forecasts. The key modeling decisions are involved in forecasting with generalized regression neural networks. For every modeling decision, several strategies are proposed. Each strategy is analyzed in terms of forecast accuracy and computational time. Apart from the modeling decisions, any successful time series forecasting methodology has to be able to capture the seasonal and trend patterns found in a time series. There are three different forecasting models proposed such as the sigmoid function regression model [9], the feedforward neural network, and the recurrent neural network model. The models were trained, compared, and validated using gas consumption data.

A novel adaptive backstepping approach is used to manage the induction motor (IM) rotor resistance tracking issue. The robustness of the device can be forecast with the experimental results. The various parameters are determined such as rotor resistance, sensitivity abd torque [10].

The genetic optimization algorithm [11] was applied to train the neural networks, and the Levenberg-Marquardt algorithm was applied to attain the parameters of the sigmoid model. From the results, it shows that both neural network models perform similarly and are superior to the sigmoid model. The models were prepared for use in conjunction with a weather forecasting service to generate day-ahead or within-day forecasts and are relevant to any geographical area.

The risk management framework is used to represent digitally the product of probability and consequence. In the conventional approach, it has been increasingly discussed to include strength of evidence combined with the traditional consequence and probability. It also focuses on addressing these challenges and makes the risk expression fully digital analysis and visualization. In the proposed approach to address the challenges by forming a fuzzy logic index based on fuzzy logic theory, this enables a transfer from a linguistic variable to a digital one. Then, it can be applied into a node size index to express its practical application. It enables an improved risk visualization, risk management, and risk communication for system analysis, towards risk digitalization.

The rule-based neuro-fuzzy approach [12] is split into two categories: the linguistic fuzzy modeling which can focus on interpretability, primarily the Mamdani model, and the fuzzy modeling that concentrated on accuracy, primarily the Sugeno model or Takagi-Sugeno-Kang (TSK) model. This rule-based approach normally applies the concept of the adaptive neural network. An adaptive network [13] is a network of nodes and directed links that is functionally equivalent to a fuzzy inference system.

In that, IF-THEN conditions are generated [14]. Individual nodes are attached with some significant parameters. The Sugeno model fuzzy rule is represented as

(1) $$\begin{array}{c} \text{IF }a\text{ is }M\text{ and }b\text{ is }N,\text{THEN }Z=f\left(a,b\right), \end{array}$$

where *M* and *N* are the fuzzy sets in the rule and “*Z*” is an output function.

This research work is arranged in this paper as follows: Section 2 describes the interrelated concepts carried out in this research domain.  Section 3 explains artificial neural network classification approach functionalities Section 4 explains the architecture and learning method of the RBFNN classifier.  Section 5 explains the step by step procedure for the proposed neuro-fuzzy approach.  Section 6 discusses the performance analysis and results, and finally, Section 7 concludes the paper.

## 2. Related Work

The fuzzy neural networks (FNN) are proposed, which have the main objective of practicing numerical relationships and practicing numerical and perception oriented information. It can reduce error rate and find the connection weights as well as bias values. A particle swarm optimization [2] is matched with the backpropagation approach for training the dataset. It produces maximum accuracy in prediction.

A novel hybrid forecasting approach [15] is based on the firefly algorithm. In that, an algorithm optimizer is combined with the adaptive neuro-fuzzy inference system for assessing the fragmentation. The proposed hybrid models were evaluated based on the statistical criteria such as coefficient of calculation and Nash and Sutcliffe. The adaptive neuro-fuzzy inference system (ANFIS) [16] is proposed to determine axial velocity and flow depth in a 90° sharp bend. The velocity and flow depth data for five discharge rates are applied for training and testing the models. In the ANFIS training phase, the two algorithms are backpropagation and a hybrid of backpropagation and least squares. In the proposed model design, the grid partitioning and subclustering methods are applied for generating the fuzzy inference system.

The fuzzy set theory [17] is used to describe an essential involvement to fuzzy concepts in data mining techniques. It manages interpretable and subjective information. A sliding window approach is used to produce time series subsequences and then analyze the fuzzy item sets. It handles temporal data to determine association rules.

The Adaptive Genetic Fuzzy System (AGFS) [18] is used for optimizing rules in the healthcare data classification. The main objective is to produce optimized rules from data. Fuzzy set theory [19] in machine learning deals with techniques for applying automated induction approaches and pattern extraction from experiential data.

A novel fuzzy partition learning approach [20] is used for applying artificial immune system methods for improving classification accuracy. An efficient CRM-data mining framework [21] is used to establish tight customer relationships and deal with the association between organizations and customers in order to take a decision. With the development of the database, the volume of data in the database increases quickly and sensitive data is protected by applying some security mechanism.

A genetic algorithm (GA) [22] is engaged to determine the optimal selection of adaptive neuro-fuzzy inference system (ANFIS) membership functions and the evolutionary design of a generalized group method of data handling (GMDH) structure for prediction of the side weir discharge coefficient. The Singular Value Decomposition (SVD) method is applied to measure the linear parameters of the ANFIS classifier and linear coefficient vectors in GMDH. The uncertainty investigation is also performed to measure the quantitative performance of all types of models.

The multilayer perceptron network [23] is applied with three types of training algorithms which include variable learning rate (MLP-GDX), resilient backpropagation (MLP-RP), and Levenberg-Marquardt (MLPLM) [23, 24]. These approaches were studied based on the ability to approximate the sediment transport in a clean pipe. Model ANN that employs volumetric sediment concentration (CV), median relative size of particles, ratio of median diameter particle size to hydraulic radius, and overall sediment friction factor as input parameters is more accurate than the other existing models.

The subfeature selection of the attributes [24] uses fuzzy methodologies to preserve privacy of the users in the distributed environment. An effective knowledge extraction approach is proposed which can get knowledge in terms of rules. At first, train the model and prune the decision tree to take out optimized rules. A correlation-oriented feature selection is introduced with a linear search approach for cardiac arrhythmia disease classification.

An adaptive neuro-fuzzy-embedded subtractive clustering (ANFIS-SC) [25] approach is applied for evaluating the abutment scour hole depth under clear water condition with uniform bed sediments. The accuracy of the ANFIS-SC approach is compared with that of two other ANFIS approaches embedded with fuzzy *C*-mean clustering [26] and grid partitioning. The decisive factors on the abutment scour hole depth include the ratio of the average diameter of particle size to abutment transverse length, excess Froude number of the abutment, shape factor, and the ratio of approach stream depth to abutment transverse length.

A genetic algorithm [27] is used for training neural networks, and analysis is made to compute the convergence error rate in a neural network. A hybrid fuzzy min-max neural network [28] is proposed, which is suitable for outlier detection. A hybrid algorithm with respect to a genetic algorithm and particle swarm optimization technique can also be applied to model a fuzzy neural network. A fuzzy wavelet neural network (FWNN) technique is another approach for obtaining better accuracy in classification.

The multilayer perceptron neural network [29] applies the artificial neural network to pick up the essential characteristics of the input layer of the network. A fuzzy radial basis polynomial network design approach [30, 31] is suitable for granular information classification. An automated healthcare classification technique [32] is introduced for wavelet transformation (WT). It is helpful in the decision support system for medical practitioners.

Neural network-based sentiment classification approaches [33, 34] such as BPNN and probabilistic NN approaches using different stages of word granularity are compared as attributes.

## 3. ANFIS Architecture

Consider the fuzzy inference method has two input values such as “*x*” and “*y*,” and “*s*” is the output. The Sugeno fuzzy method has two if-then rule constraints shown in Figure 1:

- If *x* has value *X*_1_ and *y* has value *Y*_1_, then *s*_1_ = *p*_1_*x* + *q*_1_*y* + *r*_1_
- If *x* has value *X*_2_ and *y* has value *Y*_2_, then *s*_2_ = *p*_2_*x* + *q*_2_*y* + *r*_2_

Layer 1: all the nodes are represented in

(2) $$\begin{array}{c} O_{1,i}={µX}_{i}\left(x\right),\;\text{for }i=1,2\cdots ,\\ O_{1,i}={µY}_{i-2}\left(x\right),\;\text{for }i=3,4\cdots , \end{array}$$

where “*x*” or “*y*” is the input to the node “*i*” and *X*_*i*_ (or *Y*_*i*−2_) is an associated node.

The generalized bell function is represented by

(3) $$\begin{array}{c} \mu X_{i}\left(x\right)=\frac{1}{1+{\left|\left(x-n_{i}\right)/l_{i}\right|}^{2m}}, \end{array}$$

where {*l*_*i*,_ *m*_*i*_, *n*_*i*_} is the argument set. When parameters are modified, the bell-shaped function varies consequently. These parameters are called as premise parameters.

Layer 2: in that, all the nodes are fixed. Its output is determined by finding a product of inputs. It is represented by

(4) $$\begin{array}{c} O_{2,i}=w_{i}=\mu X_{i}\left(x\right)\mu Y_{i}\left(x\right),\;\text{where }i=1,2. \end{array}$$

Layer 3: the node evaluates the proportion of the *i*^th^ rule's weighted value to the summation of the value of all weighted rules. It is denoted by

(5) $$\begin{array}{c} O_{3,i}={\bar{w}}_{i}=\frac{w_{i}}{w_{1}+w_{2}},\;i=1,2. \end{array}$$

Layer 4: in that, all nodes are adaptive in nature. It is denoted by

(6) $$\begin{array}{c} O_{4,i}={\bar{w}}_{i}f_{i}={\bar{w}}_{i}\left(l_{i}x+m_{i}y+n_{i}\right), \end{array}$$

where ${\bar{w}}_{i}$ represents a normalized weighted value of the output layer and {*l*_*i*_, *m*_*i*_, *n*_*i*_} is the consequential attribute set.

Layer 5: one node can measure the resultant value by the sum of all inputs. It is denoted by

(7) $$\begin{array}{c} \text{Output}=O_{5,1}=\underset{i}{\sum }{\bar{w}}_{i}f_{i}=\frac{\sum_{i}w_{i}f_{i}}{\sum_{i}w_{i}}. \end{array}$$

This network is the same as the Sugeno fuzzy model with respect to functionality. But structure-wise, it is different.

## 4. Radial Basis Function Networks

### 4.1. Architecture and Learning Methods

The activation stage in the hidden layer is denoted by

(8) $$\begin{array}{c} w_{i}=R_{i}\left(v\right)=R_{i}\left(\frac{\left\|x-u_{i}\right\|}{\sigma_{i}}\right),\;i=1,2,\cdots M, \end{array}$$

where “*v*” represents the input vector, *u*_*i*_ denotes the vector with the similar measurement like *v*, *M* denotes the count, and *R*_*i*_(.) is the *i*^th^ radial basis function. Weighted value have not been assigned among the input and the hidden layer shown in Figure 2.

Normally, *R*_*i*_ (.) represents the Gaussian function in

(9) $$\begin{array}{c} R_{i}\left(v\right)=\exp\left(-\frac{{\left\|v-u_{i}\right\|}^{2}}{2{\sigma^{2}}_{i}}\right). \end{array}$$

The activation stage *w*_*i*_ measured by the *i*^th^ hidden layer is greatest. In RBFN, the overall output is calculated as the weighted sum of the outputs related to the attributes. It is represented by

(10) $$\begin{array}{c} d\left(v\right)=\overset{H}{\underset{i=1}{\sum }}c_{i}w_{i}=H\overset{H}{\underset{i=1}{\sum }}c_{i}R_{i}\left(v\right), \end{array}$$

where *c*_*i*_ is represented as the connection weight between the field and the output. It is denoted in

(11) $$\begin{array}{c} d\left(v\right)=\frac{\sum_{i=1}^{H}c_{i}w_{i}}{\sum_{i=1}^{H}w_{i}}=\frac{\sum_{i=1}^{H}c_{i}R_{i}\left(v\right)}{\sum_{i=1}^{H}R_{i}\left(v\right)}. \end{array}$$

Both FIS and RBFN have a procedure whereby it can generate a center-weighted radical-shaped function. In the following constraints, an RBFN and a FIS have equal functionality:

- Both RBFN and FIS utilize the identical aggregation approach such as weighted sum and weighted average
- The receptive field unit's count in the RBFN is equivalent to the if-then rule condition in the fuzzy approach
- Subsequent radial basis function and fuzzy rule representation have similar response to the input

## 5. Proposed Method

The proposed approach can perform the selected features from a set of input prototypes, fuzzifies the equivalent prototype measures, and applies a membership function of each prototype in classes. Consider the input patterns (*N*), set of classes (*M*), and attributes (*k*). The proposed classification approach is shown in Figure 3.

The proposed technique contains three steps:

Step 1. In this fuzzification stage, a matrix order *J* × *I* is produced that contains the membership degree of *J* patterns. Every data element in this matrix is denoted as *mf*_*m*,*n*_ (*y*_*m*_), where *y*_*m*_ represents the *m*^th^ input pattern vector value, where *m* = 1, 2, ⋯, *J* and *n* = 1, 2, ⋯, *I*. The membership function is represented as

*Mf*_*m*,*n*_(*y*_*m*_) = membership pattern from class*m* to *n*, where the *m*^th^ pattern *y*_*m*_ = *x*_*m*1_, *x*_*m*2_, ⋯, *x*_*mk*_.

The input pattern vector “*y*” is represented by

(12) $$\begin{array}{c} y={\left[y_{1},y_{2},\cdots y_{J}\right]}^{T}. \end{array}$$

A generalized bell-shaped membership function is used which is based on three parameters such as *p*, *q*, and *r* as given by

(13) $$\begin{array}{c} mf\left(y:p,q,r\right)=\frac{1}{1+{\left|\left(y-r\right)/p\right|}^{2q}}. \end{array}$$

The resultant membership of the pattern vector matrix *y* is denoted by

(14) $$\begin{array}{c} MF\left(y\right)=\left[\begin{array}{ccccc} {mf}_{1,1}\left(y_{1}\right) & {mf}_{1,2}\left(y_{1}\right) & {mf}_{1,3}\left(y_{1}\right) & \cdots & {mf}_{1,I}\left(y_{1}\right)\\ {mf}_{2,1}\left(y_{2}\right) & {mf}_{2,2}\left(y_{2}\right) & {mf}_{2,3}\left(y_{2}\right) & \cdots & {mf}_{2,I}\left(y_{2}\right)\\ {mf}_{3,1}\left(y_{3}\right) & {mf}_{3,2}\left(y_{3}\right) & {mf}_{3,3}\left(y_{3}\right) & \cdots & {mf}_{3,I}\left(y_{3}\right)\\ \cdots & \cdots & \cdots & \cdots & \cdots \\ {mf}_{J,1}\left(y_{J}\right) & {mf}_{J,2}\left(y_{J}\right) & {mf}_{J,3}\left(y_{J}\right) & \cdots & {mf}_{J,I}\left(y_{J}\right) \end{array}\right], \end{array}$$

where *mf*_*m*,*n*_ (*y*_*m*_) is the member of *m*^th^ pattern of input values “*y*” where *m* = 1, 2, ⋯, *J*.

Step 2. In this step, MLPBPN is constructed. It converts the matrix values into an *M* × *N* vector by transposing it. This converted vector value is applied as input to the classifier.

A distinctive MLPBPN approach has a one input and output layer and a minimum one hidden layer. It demonstrates two types of procedures: feedforward and backpropagation. The nodes are associated in a feedforward approach. The input nodes are linked to the hidden nodes, and the hidden elements are entirely related to the output layer elements. The input and hidden nodes are linked with the weighted value. All weighted values of nodes are preferred arbitrarily shown in Figure 4.

In the backpropagation method, the happening of errors and the learning process such as revising the weighted value and biases are transmitted in the reverse route beginning from the output level to the internal values. This procedure is replicated many times. The main objective is to reduce the root-mean-square error among the forecast and actual values up to completion of the preparation process or the final condition attained [35–39].

The predicted output of element “*n*” is represented by

(15) $$\begin{array}{c} {\text{Output}}_{n}=\frac{1}{1+e^{-{\text{Net}}_{m}}}, \end{array}$$

where Net_*n*_ is the total input of element “*n*” in this model. The total input value is represented as a sum of the connection strengths and the result from the previous stage. It is represented in

(16) $$\begin{array}{c} {\text{Net}}_{n}=\underset{m}{\sum }{\text{weight}}_{m,n}\times {\text{Output}}_{m}+{\text{bias}}_{n}, \end{array}$$

where weight_*m*,*n*_ is the connection strength of the connection from element “*m*” in the preceding stage to unit “*n*.” Output_*m*_ is the output of element “*m*” from the previous stage, and bias_*m*_ is the bias of the element.

The total of squared error values from the predictable result is measured by

(17) $$\begin{array}{c} \text{Error}=\frac{1}{2}\underset{n}{\sum }{\left({\text{Target}}_{n}-{\text{Output}}_{n}\right)}^{2}. \end{array}$$

The weighted value of the backpropagation network model is changed to decrease this error. It is denoted in

(18) $$\begin{array}{c} \Delta \text{Weight}\infty -\frac{\partial \text{Error}}{\partial \text{Weight}}. \end{array}$$

The final output stage “*n*” with a weight value, weight_*m*,*n*_, is determined by

(19) $$\begin{array}{c} \Delta {\text{Weight}}_{m,n}\infty -\frac{\partial \text{Error}}{\partial {\text{Weight}}_{m,n}},\\ \Delta {\text{Weight}}_{m,n}=-\eta \frac{\partial \text{Error}}{\partial {\text{Output}}_{n}}\times \frac{\partial {\text{Output}}_{n}}{\partial {\text{Net}}_{n}}\times \frac{\partial {\text{Net}}_{n}}{\partial {\text{Weight}}_{m,n}}, \end{array}$$

where *η* denotes the learning rate. Here, the weight updating formula is represented as

(20) $$\begin{array}{c} {\text{Weight}}_{m,n}={\text{Weight}}_{m,n}+\Delta {\text{Weight}}_{m,n}. \end{array}$$

Similarly, bias updation is performed by

(21) $$\begin{array}{c} {\text{bias}}_{n}={\text{bias}}_{n}+\Delta {\text{bias}}_{n}. \end{array}$$

In the MLPBPN approach, only one hidden layer is used. The neural network approach uses gradient descent with impetus as supervised conditions. Both hidden and last layers follow the tan sigmoidal transfer function.

The input layer nodes are equivalent to the amount of input features in the datasets. In the same way, the count of resultant nodes is equal to the quantity of class labels. The elements in the hidden layer are denoted as *L* in

(22) $$\begin{array}{c} L=\left(\text{Input featurecount}+\text{Total classcount}\right)*\frac{2}{3}. \end{array}$$

Step 3. In this defuzzification stage, the proposed classifier classifies and defuzzifies the activation result. The input prototype is selected to the class “*n*” with the highest membership label.

### 5.1. Detailed Procedure

(Step 1) Apply data cleaning in which preprocessing of data is performed by eliminating or decreasing noise. The attribute missing values are replaced by its mean value.
(Step 2) Apply data selection in which statistical correlation analysis is applied to remove duplicate features, and then, only the relevant features can be collected.
(Step 3) Apply transformation of data in which normalization is applied to the dataset. The neural network-based technique involves transformation of values ranging from −1.0 to +1.0.
(Step 4) The data is separated into two subsets, training and test datasets, after preprocessing.
(Step 5) In the training stage, the data is applied to the proposed system for creating a prototype. It also implemented for both RBFNN and ANFIS approaches for developing other classifiers.
(Step 6) In the testing stage, three classifiers such as NFS, RBFNN, and ANFIS are applied for calculating its performance.
(Step 7) The performance measures of these models are compared.

The detailed procedure is shown in Figure 5.

## 6. Results and Analysis

In our experiment, three classification approaches such as HNFC, RBFNN, and ANFIS are applied on benchmark datasets, namely, primary tumor, breast cancer, *E. coli*, mushroom, diabetes, ionosphere, liver disorder, Credit-g, Anneal-org, and iris. From the machine learning repository using the R tool, there are 50,000 records that are created for each dataset and compare its performance. In the breast cancer dataset, it has ten numbers of features such as age, mefalsepause, tumor size, inv-falsedes, falsede-caps, deg-malig, breast, breast-quad, and irradiat. All the features are multivariate categorical type of attributes.

A performance comparison has been done by considering various metrics such as accuracy, TP-rate, FP-rate, precision, *F*-measure, and root mean square error (RMSE). From the experimental outcomes given in Table 1, for the above specified datasets, the proposed HNFC method has produced better classification accuracy compared to other two approaches such as RBFNN and ANFIS.

### 6.1. Performance Measures

The performances of the classifiers are evaluated as per the following metrics:

#### 6.1.1. Confusion Matrix

The confusion matrix is an illustration which gives the detailed visualization of the classification performance. Each column represents the records in a predicted variable. The row denotes the records in an actual variable.

- True positive is a count of correct and positively classified objects
- False positive is a count of incorrectly classified instances which are positive
- False negative is a count of incorrectly classified instances which are negative
- True negative is a count of correctly classified objects that are negative

Accuracy of the correctly classified instance is determined by

(23) $$\begin{array}{c} \text{accuracy}=\frac{\text{tp}+\text{tn}}{\text{tp}+\text{tn}+\text{fp}+\text{fn}}. \end{array}$$

The relation of the forecast positive objects which are accurate is determined by

(24) $$\begin{array}{c} \text{Precision}=\frac{\text{tp}}{\text{tp}+\text{fp}}. \end{array}$$

The relation of negative objects which are incorrectly classified as positive is represented by

(25) $$\begin{array}{c} \text{FP}‐\text{rate}=\frac{\text{fp}}{\text{fp}+\text{tn}}. \end{array}$$

The relation of positive objects which are suitably classified is calculated by

(26) $$\begin{array}{c} \text{recall}=\text{tp}‐\text{rate}=\frac{\text{tp}}{\text{tp}+\text{tn}}. \end{array}$$

In some situations, maximum recall value may be important. To increase the performance measures, both precision recall values are represented by

(27) $$\begin{array}{c} F‐\text{measure}=\frac{2*\text{precision}*\text{recall}}{\text{precision}+\text{recall}}. \end{array}$$

From Table 2, while the breast cancer dataset is taken as input and applied to existing classifiers such as RBFNN and ANFIS, it produces the accuracy of 83.3% and 82.2%, respectively. But at the same time, for the proposed hybrid neuro-fuzzy classification, it gives 86.2%. It is comparatively higher than that of the other two approaches. Root mean square error is also low (0.323) for the proposed system. Time complexity is high compared to that of other decision tree classification approaches. But this drawback can be overcome by means of producing maximum accuracy in classifications. The existing approaches with the proposed algorithms have been applied for other datasets such as diabetes, liver disorder, E. coli, primary tumor, mushroom, ionosphere, Credit-g, Anneal-org, and iris. The performance comparison has been shown in Figures 6 and 7.

Figure 8 denotes the various features of the breast cancer dataset and relationship among various data items in the dataset. Red color circle denotes the recurrence events, and blue color denotes no recurrent events in the dataset.

From the above experimental graphs, for the breast cancer dataset, a number of instances are distributed and the class labels are indicated in red and blue color circle format. With respect to various attribute values, the distribution ranges and values will be varied. The chart representation indicates the accuracy for the various existing algorithms such as the radial basis function neural network and adaptive network-based fuzzy inference system; the proposed hybrid neuro-fuzzy classifier provides better classification accuracy for the various input data such as breast cancer, diabetes, E. coli, liver disorder, primary tumor, mushroom, ionosphere, Credit-g, Anneal-org, and iris.

## 7. Conclusion

In this paper, we compared the proposed HNFC approach with RBFNN and ANFIS classification. The classifiers were experimented with ten UCI repository datasets. From the experimental outcome, the proposed classifier produces 86.2% better performance in classification of datasets compared to the existing algorithms. Similarly, this classifier provides better performance in classifying the input data. And it also provides a valuable contribution to the performance improvement of conventional classification approaches in the data mining research field. Still there is a research opening to apply other classifiers to predict the disease based the medical records.

## Figures and Tables

**Figure 1:** ANFIS architecture layer-wise representation.

**Figure 2:** Input, hidden, and output layer of the RBFNN model.

**Figure 3:** Proposed neuro-fuzzy classification approach.

**Figure 4:** MLPBPN architecture layer-wise procedure.

**Figure 5:** Detailed steps for the development of the proposed system.

**Figure 6:** Performance measures for the breast cancer dataset.

**Figure 7:** Comparison of classification accuracy for various datasets.

**Figure 8:** Distribution and recurrent relationship among features in the dataset.

**Table 1:** List of features of the breast cancer dataset.

S. no	List of attributes	Type of data
1	Age	Numeric
2	Mefalsepause	Numeric
3	Tumor size	Numeric
4	Inv-falsedes	Numeric
5	Falsede-caps	Numeric
6	Deg-malig	Numeric
7	Breast quad	Numeric
8	Irradiat	Numeric
9	Class	Categorical

**Table 2:** Detailed performance comparison for three classifiers.

Datasets	Classifiers	Acc (%)	TP rate/recall (%)	FP rate (%)	Precision (%)	*F*-measure (%)	TT (sec)
Breast cancer	HNFC	86.2	85.2	14.8	85.5	85.2	1521.2
	RBFNN	83.3	82.3	17.7	82.8	82.3	1821.5
	ANFIS	82.2	80.5	19.5	82.1	80.5	1712.2

Diabetes	HNFC	85.4	83.5	16.5	82.6	83.5	1514.6
	RBFNN	80.4	78.6	21.4	79.6	78.6	1815.2
	ANFIS	79.2	77.5	22.5	78.5	77.5	1945.2

E. coli	HNFC	75.9	74.2	25.3	76.5	74.2	1612.2
	RBFNN	73.6	72.8	27.2	71.6	72.8	1812.2
	ANFIS	72.8	71.5	28.5	72.1	71.5	1921.2

Liver disorder	HNFC	78.8	77.8	22.2	77.8	77.8	1621.2
	RBFNN	76.8	74.5	25.5	74.5	74.5	1752.6
	ANFIS	70.2	71.5	28.5	71.5	71.5	1721.6

Primary tumor	HNFC	80.4	80.2	19.8	78.5	80.2	1825.5
	RBFNN	78.6	77.3	22.7	75.6	77.3	2112.5
	ANFIS	77.6	75.8	24.2	72.8	75.8	2512.6

Mushroom	HNFC	92.5	91.1	8.9	90.5	91.1	1321.2
	RBFNN	90.6	88.5	11.5	89.5	88.5	1521.9
	ANFIS	88.9	87.8	12.2	87.2	87.8	1569.3

Ionosphere	HNFC	95.5	94.1	5.9	93.5	94.1	1125.6
	RBFNN	93.6	92.5	7.5	91.3	92.5	1253.2
	ANFIS	92.2	90.1	9.9	89.6	90.1	1245.6

Credit-g	HNFC	96.8	94.6	5.4	89.5	94.6	1325.2
	RBFNN	93.8	92.2	7.8	90.6	92.2	1452.2
	ANFIS	91.8	90.8	9.2	89.9	90.8	1441.3

Anneal-org	HNFC	95.9	94.8	5.2	93.5	94.8	1221.2
	RBFNN	93.8	92.5	7.5	91.8	92.5	1362.3
	ANFIS	91.5	90.6	9.4	90.6	90.6	1401.2

Iris	HNFC	96.8	95.6	4.4	95.2	95.6	1323.1
	RBFNN	94.2	94.1	5.9	93.6	94.1	1391.2
	ANFIS	93.5	92.5	7.5	90.8	92.5	1423.2

## Data Availability

The data used to support the findings of this study are included in the article.
